# PDNet: Improved YOLOv5 Nondeformable Disease Detection Network for Asphalt Pavement

**DOI:** 10.1155/2022/5133543

**Published:** 2022-07-07

**Authors:** Zhen Yang, Lin Li, Wenting Luo

**Affiliations:** ^1^College of Transportation and Civil Engineering, Fujian Agriculture and Forestry University, Fuzhou, Fujian 350108, China; ^2^College of Transportation Engineering, Nanjing Tech University, Nanjing, Jiangsu 211816, China

## Abstract

In the daily inspection task of the expressway, accuracy and speed are the two most important indexes to reflect the detection efficiency of nondeformation diseases of asphalt pavement. To achieve model compression, accelerated detection, and accurate identification under multiscale conditions, a lightweight algorithm (PDNet) based on improved YOLOv5 is proposed. The algorithm is improved based on the network structure of YOLOv5, and the improved network structure is called YOLO-W. Firstly, a novel cross-layer weighted cascade aggregation network (W-PAN) is proposed to replace the original YOLOv5 network. Secondly, more economical GhostC3 and ShuffleConv modules are designed to replace C3 and Conv modules in the original network model. In terms of parameter setting, CIoU is selected as the loss function of the model, and the K-Means ++ algorithm is used for anchor box clustering. Before the model training, the confrontation generation network (GAN) and Poisson migration fusion algorithm (Poisson) are used for data enhancement and the negative sample training (NST) method is used to improve the robustness of the model. Finally, Softer-NMS is used to remove the prediction box in the prediction stage. Seven common asphalt pavement disease data sets (FAFU-PD) are constructed at the same time. Compared with the original YOLOv5 algorithm, PDNet improves the scores of FAFU-PD data sets on F1-score by 10 percentage points and FPS by 77.5%.

## 1. Introduction

Asphalt pavements on expressways are damaged by natural disasters, such as prolonged exposure to sunlight, rain erosion, and natural weathering. And the durability of asphalt pavement will also be reduced due to factors such as pavement materials, traffic flow, construction quality, and postmaintenance levels. If these damaged roads cannot be discovered and maintained in time, the service life of the expressway will be shortened, which may induce traffic accidents [1].

At present, the detection of highway asphalt pavement diseases is mainly based on manual methods. This method has some disadvantages. For example, the detection takes a long time and requires more manpower and material resources, and the detection will cause congestion on the highway, and the safety of the detection personnel is difficult to be guaranteed. At the same time, some human factors interfere with the test results. With the continuous increase of highway mileage, manual detection methods are difficult to meet the detection requirements of large-scale highways and cannot meet the needs of highway development [2].

To further improve the service life of highways and use an accurate and efficient detection method to replace the traditional manual detection method, some researchers have conducted research on the automatic detection of pavement diseases based on visual technology, which includes image processing, machine learning, and deep learning. Image processing research includes threshold segmentation, edge detection, and regional growth. The threshold segmentation method is mainly to set the appropriate pixel threshold in the image and separate the disease from the background by using the pixel difference between the crack and the surrounding background. The edge detection method mainly realizes the edge detection through various edge detection operators. These edge detection operators include Sobel operator [3], Prewitt operator [4], and Canny operator [5]. The region growing method mainly displays the specific information inside the disease through pixel integration.

Compared with the traditional manual detection method, the image processing method has been greatly improved, but this method is easily disturbed by external factors such as road background and sunlight, the types of road diseases are complex and diverse, and the image processing method is difficult to detect various types of complex diseases [6].

In recent years, machine learning and deep learning have developed rapidly, especially in industrial applications. It has become possible to use machine learning or deep learning to build a model for pavement disease detection. Machine learning methods mainly include wavelet transform, support vector machine, and random forest methods. Among the deep learning methods, convolutional neural networks (CNNs) have made great progress in semantic segmentation and target detection tasks. From the current development status of the target detection field, the target detection methods based on deep learning are mainly divided into one-stage method and two-stage method. The two-stage method mainly includes R-CNN [7], fast-RCNN [8], and faster-RCNN [9]. The advantages of these algorithms are high recognition accuracy, but they also have the disadvantage of slow speed, so it is not suitable for engineering applications. To solve this shortcoming of the two-stage method, the researchers proposed the algorithm framework of the one-stage method. The representative works include SSD [10], YOLO series, and anchor-based RetinaNet [11], Adaptive Sample Selection (ATSS) [12], Fully Convolutional One-Stage Object Detection (FCOS) [13], and Anchor-Free Based RepPoints [14].

At present, whether it is based on traditional image processing methods or methods based on machine learning and deep learning, there are still some problems in the detection of asphalt pavement diseases: (1) based on traditional image processing methods, in terms of recognition speed, the effect is poor, and it is difficult to deal with complex engineering tasks. (2) The cost of network training and prediction using machine learning and deep learning methods is too high, and the use of feature extraction will make the network lose real-time performance and cannot meet industrial needs. (3) The engineering application scenarios are complex, and there are various types of diseases, and it is difficult to guarantee the accuracy and recall rate of disease identification. Figures 1(a) and 1(b) are schematic diagrams of the redundancy of the target frame; Figures 1(c) and 1(d) show that the model incorrectly identifies negative samples as positive samples; Figures 1(e) and 1(f) show a schematic diagram of inaccurate prediction of anchor boxes; Figures 1(g) and 1(h) show the situation that the model does not extract disease features in place. (4) There is a lack of large data sets for various types of diseases.

To meet the real-time performance and improve the accuracy and recall rate of target recognition, this study proposes a real-time, lightweight, and higher-precision target detection algorithm (PDNet) based on YOLOv5. In Section 2, this article mainly introduces the domestic and foreign research status of nondeformation disease detection of asphalt pavement, and Section 3 introduces the research methods used in this article.  Section 3.1 introduces the overall architecture of the YOLO-W network proposed in this article; Section 3.2 introduces the cross-layer weighted cascade aggregation network (W-PAN); Section 3.3 introduces the improved GhostC3 module; Section 3.4 introduces the improved ShuffleConv module; Section 3.5 is mainly about the settings of network model parameters, including loss function and anchor frame settings, respectively; Section 3.6 introduces a data set of seven diseases including transverse cracks, longitudinal cracks, and repair strips collected from one province and four cities (FAFU-PD); Section 3.7 introduces a negative sample algorithm (NST) for the problem of model misidentification, which can effectively improve the recognition accuracy of the model; Section 3.8 uses an adversarial generative network (GAN) to generate a larger number of samples; Section 3.9 uses the Poisson transfer fusion algorithm, which is transplanted based on GAN to generate disease-free pictures to generate new disease samples; Section 3.10 introduces the Softer-NMS algorithm. It solves the problem that there are many false detections of diseases in dense scenes and the positioning of the prediction frame with high default confidence of NMS is not very accurate.  Section 4 is the experimental part, Section 4.1 introduces the data and experimental environment used in this experiment, and Section 4.2 is the ablation experiment for each method proposed in Section 3.  Section 5 analyzes the methods proposed in this article and describes the advantages of each method.  Section 6 summarizes this article.

The main contributions of this article are as follows:

1. It proposes an improved target detection network YOLO-W. First, to prevent the loss of shallow target features, a cross-layer cascaded weighted fusion structure is added to the PANet structure to transfer detailed information to the deep network, and a cross-layer weighted cascaded path aggregation network (W-PAN) is proposed to obtain richer semantic information, deepen the depth of the pyramid, correspondingly increase the detection layer of the head part, and perform detection at four scales, so that the laying interval of anchor boxes is more reasonable; finally, it reduces the feature loss caused by the upsampling process, which improves the upsampling method.
2. Lightweight network: the GhostC3 module is used to replace the original C3 module, and the ShuffleConv module is used to replace part of the Conv module, which alleviates the problem of computational occupancy in the process of feature channel fusion and enhances the expressiveness of features.
3. uses the K-Means ++ algorithm to redesign the size of the prior box and match it to the corresponding feature layer.
4. The negative sample training method (NSTM) is adopted to improve the detection accuracy without reducing the detection speed and reduce the false detection rate.
5. uses an adversarial generative network (GAN) to generate diseases with a small number of samples.
6. uses the Poisson transfer fusion algorithm to transfer the color of the sample generation disease to make it better match the sample and add the generated sample to the training set and the validation set.
7. constructs 7000 data sets (FAFU-PD) including one province, four cities, and seven diseases.

## 2. Related Studies

### 2.1. Pavement Damage Detection Method Based on Image Processing and Machine Learning

In the early days, most of the pavement disease detection methods based on image processing [15–17] were based on threshold segmentation, because, in images with cracks and other diseases, the pixel values of cracks and diseases are darker than the surrounding background, and threshold segmentation is used. The contours of diseases such as cracks can be well extracted. Early researchers proposed crack detection algorithms based on threshold segmentation from different perspectives. Oliveira and Correia [18] proposed a new framework for automatic crack detection and classification. This framework preprocesses the generated images using morphological filters to reduce pixel intensity variations. Then, dynamic thresholding was applied to identify dark pixels in the image, and a second dynamic threshold was applied to the resulting matrix of entropy blocks, which was used as a basis for identifying image blocks containing cracked pixels. Ayenu-Prah and Attoh-Okine used BEMD and Sobel edge operators for pavement crack detection. Multiple images were filtered by BEMD to remove noise, and the residual image was analyzed by Sobel edge operator [19]. Yan et al. introduced morphology into crack detection of high-grade highway pavement and proposed a new image processing method. This method reconstructs the median filter algorithm to enhance the pavement grayscale image and combines the morphological gradient operator and the morphological closure operator to extract crack edges and fill crack gaps [20]. Wei et al. proposed a pavement crack detection algorithm based on Beamlet transform [21]. Wavelet transform is also one of the common methods for pavement crack detection [22–24]. However, the above methods are very susceptible to noise interference, and it is difficult to obtain accurate detection results. Nguyen et al. proposed a new method that considers both brightness and connectivity in the segmentation step for crack detection in road surface images. Features computed along each free path can detect cracks in any form and any direction [25]. Amhaz et al. proposed a new algorithm for automatic crack detection from 2D road surface images. This algorithm, which relies on the localization of the smallest path in each image, has been intensively validated on synthetic and real images, and it provides very stable and accurate results in a variety of situations in a completely unsupervised manner [26]. Ai et al. proposed a new method to automatically detect pixel-level pavement cracks using multiscale neighborhood information and pixel intensities. Using the pixel intensity information, a probabilistic generative model (PGM) based method was developed to calculate the crack presence probability for each pixel [27]. Shi et al. introduced random structure forests to generate high-performance crack detectors that can identify arbitrarily complex cracks [28]. However, these traditional methods rely heavily on postprocessing and require a large amount of computation, which is not conducive to engineering applications.

### 2.2. Pavement Damage Detection Method Based on Deep Learning

In recent years, the application of deep learning methods in the field of target detection has become more and more extensive, including the identification of nondeformable diseases of asphalt pavement. Neural networks such as CNN and R-CNN have played an important role in the field of target detection. Cha et al. proposed a vision-based approach that uses a deep architecture of convolutional neural networks (CNNs) to detect cracks without computing defect features. Since CNN can learn image features automatically, the proposed method can extract features without IPT conjugation [29]. Zhang et al. used CNN convolutional neural network for image preclassification [30]. Yang et al. implemented a novel deep learning technique called a fully convolutional network (FCN) to solve the pixel-level crack identification problem [31]. Chen and Jahanshahi proposed a deep learning framework based on convolutional neural network (CNN) and a naive Bayesian data fusion scheme called NB-CNN for analyzing a single video frame for crack detection and proposed a new data fusion scheme is proposed to aggregate information to improve the overall performance and robustness of the system [32]. Park et al. proposed a CNN-based deep learning model, patch-CNN, which consists of segmentation and classification modules for crack detection [33]. Zou et al. proposed an end-to-end trainable deep convolutional neural network (DeepCrack) for automatic crack detection by learning high-level features represented by cracks [34]. These deep learning-based methods can improve the accuracy of disease identification to a certain extent, but they cannot achieve both recognition speed and accuracy and lose speed while improving the accuracy of disease identification.

## 3. Methodology

Figure 2 shows the overall network structure of the algorithm (PDNet) shown in this article. In the preprocessing stage, a generative adversarial network (GAN) is used to generate a small number of disease types, and then the Poisson color transfer algorithm is used to generate the generated diseases. The image is fused with the background to obtain new disease samples. Secondly, all negative samples that are prone to misidentification are labeled (NST). After processing, all training and validation sets are sent to the training network (YOLO-W). At the prediction end, the Softer-NMS algorithm is used to remove redundant boxes to obtain the final recognition result.

### 3.1. The Overall Architecture of the YOLO-W Network

YOLO-W is a high-performance target detection network based on YOLOv5. It adopts a cross-layer weighted cascaded path aggregation network (W-PAN) to improve the accuracy of model recognition and lightweight modules GhostC3 and ShuffleConv to reduce the complexity of the network. The network structure of YOLO-W is shown in Table 1. The changes in the backbone and neck parts of YOLO-W compared with the original YOLOv5 network model are shown in Figures 3 and 4.

Among them, “from” represents the output layer corresponding to this layer module, and “−1” represents the previous layer. “Add” represents the cross-layer weighted addition module in W-PAN, and “GhostC3” and “ShuffleConv” represent the GhostC3 module and ShuffleConv module used in YOLO-W, respectively.

### 3.2. Cross-Layer Weighted Cascade Aggregation Network (W-PAN)

The shallow network of deep learning focuses on detailed information, such as edge features. Based on obtaining simple features, it can help the network return to the target boundary more accurately; the deep network focuses on extracting high-level semantic information and can extract more complex features, which can help the network detect the target accurately. The FPN structure uses shallow features to distinguish simple objects and deep features to distinguish complex objects, aiming to obtain more robust detection results. The FPN structure of YOLOv5 is based on PAN, which creates a bottom-up path enhancement, accelerates the flow of underlying information, and can well integrate semantic information at all levels. To further enhance the model's attention to shallow semantics, fully integrate the semantic information extracted by each layer of the FPN, and enhance the network's ability of returning to the target boundary, this study improves the FPN of YOLOv5, called W-PAN, and the specific improvement points are as follows:

(1) Add cross-layer weighted connections between input and output nodes of the same size [35]. The cross-layer cascade structure can effectively integrate the shallow details, edges, contours, and other information into the deep network and can fuse the shallow details of the target with almost no increase in the amount of calculation so that the network can be more sensitive to the target boundary. The regression is more accurate, and the intersection ratio between the predicted frame and the real frame is effectively improved. At the same time, considering that the integration of shallow features will have a certain impact on deep semantic information when using cross-level concatenation, a learnable method is adopted for fusion. The two fusion methods used in this study are given as follows: in the process of feature fusion, since the information flow of the top and bottom nodes is fast and the number of convolutions experienced is small, the loss of detailed information is not much. There is complexity of the small model, so the concat operation is directly used to perform feature fusion by channel. The process is shown in Figure 5. *F* represents the feature map, *w* represents the width of the feature map, *h* represents the height of the feature map, and *c* represents the number of channels of the feature map.
For nodes in other layers, the concat operation is used for feature fusion on adjacent paths, and the weighted add operation with learnable weights is used for feature fusion on nonadjacent paths. The add operation can not only reduce the amount of calculation but also reduce the amount of invalid shallow information. Fusion calculation is shown in the following formula:
  (1) $$\begin{array}{c} \text{OUT}=\sum_{i}\frac{\mu_{i}\cdot x_{i}}{\varepsilon +\sum_{j}\mu_{j}}, \end{array}$$
where *x*_*i*_ represents each feature map to be fused; *?* is the weight coefficient of the feature map, which can be updated through learning. The initial weight coefficient is set to 1, indicating that the two layers of feature maps are fused equally; *ε* is a very small number (≤10^−3^) which can effectively prevent numerical instability. Normalizing the weights between 0 and 1 increases the speed of training while preventing unstable training. According to formula (1), the feature fusion method for an intermediate layer is shown in Figure 6.
In Figures 5 and 6, given the input feature map *F*_1_ ∈ *ℝ*^*w*×*h*×*c*_1_^ of a certain layer, the top-down path corresponds to the layer's feature map *F*_2_ ∈ *ℝ*^*w*×*h*×*c*_2_^, and the bottom-up path corresponds to the layer's feature map *F*_3_ ∈ *ℝ*^*w*×*h*×*c*_3_^, “*∗*” indicates the concat operation, “+” indicates the add operation, and weight1 and weight2 are the weight values of the feature map fusion on the two paths, respectively. It can be seen from the two figures that the feature fusion of the top and bottom output nodes adopts the concat operation, while the feature fusion of the middle layer nodes first undergoes the concat operation and then performs weighted add with the channel-aligned input layer operation. The final feature map obtained at the output node is a composite feature map containing details, edges, and high-level semantic information. For ease of understanding, taking the middle layer P4 as an example, the calculation of the output on each path is shown in the following formulas:
  (2) $$\begin{array}{c} P4^{\mathrm{td}}=\text{Concat}\left(P4^{\mathrm{in}},\text{Resize}\left(Conv\left(P5^{\text{in}}\right)\right)\right), \end{array}$$
  (3) $$\begin{array}{c} P4^{\mathrm{out}}=\frac{\mu_{1}\cdot \text{Concat}\left(P4^{\mathrm{td}},\text{Resize}\left(Conv\left(P3^{\mathrm{out}}\right)\right)\right)+\mu_{2}\cdot P3^{\text{out}}}{\varepsilon +\mu_{1}+\mu_{2}}, \end{array}$$
where *Pk*^*in*^ represents the input of the kth layer, *Pk*^*td*^ represents the output of the kth layer intermediate node in the top-down path, and *Pk*^out^ represents the output of the kth layer output node in the bottom-up path.
(2) Increase the depth of the feature pyramid upwards. The high-level perception field of FPN is large, and the semantic information contained is more advanced, which can increase the learning ability of the network and further improve the detection accuracy. The FPN of YOLOv5 is 3 layers. Based on improvement 1, this study deepens it to 4 layers, which can make full use of the proposed cross-layer cascade structure. In addition, to match the depth of FPN, this study adds the detection layers of the detect part, named tiny, small, medium, and large, respectively, performs target detection on the feature maps output by P3, P4, P5, and P6 in turn, and increases the detection. The laying interval of anchor boxes after the layer becomes more reasonable, and the stability of training and the convergence speed and accuracy of the model will be effectively improved. Based on the improvement points 1 and 2, the simplified version of the FPN structure used in this article is shown in Figure 7.
The red dotted line in Figure 7 is the cross-layer cascading. It can be seen from the figure that the cross-layer weighted fusion is only used for the two middle layers P4 and P5. For the top layer P6 and the bottom layer P3, there is no much loss due to information flow. Considering the operating efficiency of the model, this study directly splices the two feature maps by channel. To objectively give the impact of deepening the pyramid on the network, Table 2 shows the comparison of the effect of YOLOv5s before and after deepening the pyramid, where W-PAN-Deep represents the PAN module after deepening the pyramid.
The comparison of the effect of YOLOv5s before and after deepening the pyramid shows that, after deepening the pyramid, although the F1-score of the model has been greatly improved, the large increase in the number of parameters makes loading the network need more video memory, which not only increases the hardware requirements for model training but also affects the speed at which the model runs. To solve such a problem, this study introduces the Ghost series of modules to lighten the network, to a certain extent, to make up for the negative impact of the increased network complexity after deepening the pyramid.
(3) Improve the YOLOv5 upsampling method. YOLOv5 uses the nearest neighbor interpolation method for upsampling. This method uses a single reference point pixel value for estimation. Although the speed is fast and the overhead is small, the upsampling process will cause serious feature loss and reduce the detection accuracy of small targets. The bilinear interpolation method uses four points to estimate the interpolation, and the obtained feature map is more delicate and the loss of details is less. Therefore, this study changed the upsampling method to the bilinear interpolation method, and the complexity of the two is only a constant level gap, relatively to the improvement in accuracy; the computational overhead is acceptable.  Table 3 shows the experimental accuracy comparison of YOLOv5s using PAN structure and two W-PAN structures; W-PAN indicates that the FPN structure proposed in this study is completely used.

It can be seen from the table that the F1-score index of using W-PAN is improved by 5.16% compared with that of PAN and the F1-score index of W-PAN-Deep, which deepens the pyramid, is improved by 1.6%, which proves that the cross-level cascade structure can further improve the regression accuracy of the network to the boundary. In general, the W-PAN structure makes the fusion of semantic information at all levels of the network more reasonable and sufficient. The introduction of W-PAN has greatly improved the accuracy of the network, especially the accuracy of high intersection and is higher than the required accuracy, which proves that the network from The W-PAN structure incorporates more effective feature information, which can better return the bounding box of the target and fit the industrial target detection task of high cross-comparison.

### 3.3. Improved GhostBottleneckCSP

GhostNet proposes an innovative module Ghost, which generates more feature maps with fewer parameters and computations [36]. The implementation of Ghost is divided into 2 parts, one is ordinary convolution, and the other is a linear operation with fewer parameters and computations. First, a part of the feature map is obtained through limited ordinary convolution, and then the obtained feature map is linearly operated to generate more feature maps, and finally the two sets of feature maps are spliced in the specified dimension. The operating principle of Ghost is shown in Figure 8.

The operation of the ordinary convolution layer is shown in

(4) $$\begin{array}{c} Y=X*f+b. \end{array}$$

The Ghost module containing block contains a small number of convolutions, a population identity map, and *m* × (*s* − 1) linear operations. First, generate a small number of feature maps through general convolution; then perform cheap linear operations on the feature maps obtained in the first step to generate Ghost feature maps. Finally, the two sets of feature maps are spliced by channel to generate enough feature maps to match the given number of output channels.

For an input *X* ∈ *ℝ*^*W*×*H*×*C*^, the output *Y* ∈ *ℝ*^*W*′×*H*′×*n*^ of a general convolution can be denoted by *Y*=*X* · *f*+*b*, the *f* ∈ *ℝ*^*k*×*k*×*C*×*n*^ represents *C* × *n* convolution operations with a kernel size of *k* × *k*, and *b* represents the bias term. *W* and *H* represent the width and height of the input feature map, respectively. *W*′ and *H*′ represent the width and height of the output feature map, respectively. *C* refers to the number of input channels. The FLOPs of a general convolution can be denoted by *W*′ · *H*′ · *n* · *k* · *k* · *C*. Ghost convolution adopts the step-by-step strategy, and the calculation method is shown in

(5) $$\begin{array}{c} Y^{\prime }=X\cdot f^{\prime }, \end{array}$$

(6) $$\begin{array}{c} Y_{ij}=\Phi_{ij}\cdot Y_{i}^{\prime },i\in \left[1,m\right],\;j\in \left[1,s\right]. \end{array}$$

In a small number of convolution results, *Y* ∈ *ℝ*^*W*′×*H*′×*m*^ represent the *m* feature maps (*m* ≪ *n*) generated by the general convolution *f*′ ∈ *ℝ*^*k*×*k*×*C*×*m*^ on the input *X*; then the *m* feature maps are linearly operated one by one, and each feature map generates *s* feature maps, and a total of *n*=*m* × *s* feature maps are generated. Feature map Φ_*ij*_ represents the *ith* linear operation on the *jth* feature map *Y*_*i*_′ generated in the first step of convolution; Φ_*i*,*s*_ represents a direct feature identity map. To ensure the efficiency and practicability of CPU or GPU, set the size of the convolution kernel of each linear operation to be *d* × *d*; then the speed ratio of general convolution and Ghost convolution can be calculated by

(7) $$\begin{array}{c} RATE_{s}=\frac{W^{\prime }\cdot H^{\prime }\cdot n\cdot k\cdot k\cdot C}{W^{\prime }\cdot H^{\prime }\cdot m\cdot k\cdot k\cdot C+W^{\prime }\cdot H^{\prime }\cdot \left(n-m\right)\cdot d\cdot d\cdot C}\\ =\frac{W^{\prime }\cdot H^{\prime }\cdot n\cdot k\cdot k\cdot C}{W^{\prime }\cdot H^{\prime }\cdot \left(n/s\right)\cdot k\cdot k\cdot C+W^{\prime }\cdot H^{\prime }\cdot \left(s-1\right)\cdot \left(n/s\right)\cdot d\cdot d\cdot }\\ =\frac{k\cdot k\cdot C}{\left(1/s\right)\cdot k\cdot k\cdot C+\left(\left(s-1\right)/s\right)\cdot d\cdot d}\\ \approx \frac{s\cdot C}{s+C-1}\\ \approx s. \end{array}$$

Here, *k* × *k* and *d* × *d* have the same size, and *s* ≪ *C*. From the simplification results, the calculation amount of general convolution is roughly *s* times that of Ghost convolution. Similarly, the number of parameters can be calculated as *s* times. Ghost convolution is a lighter and faster module. Based on this, this study designs GhostBottleneck and GhostBottleneckCSP modules based on the Ghost module. The specific structure is shown in Figure 9.

*C*_1_ and *C*_2_ in Figure 9 refer to the number of channels of input and output characteristic graphs, respectively. In this article, the 1 × 1 ordinary convolution shown in Figure 9(a) is used to reduce the number of channels to 1/2 of the number of output channels, and then a depthwise convolution with a size of 5 × 5 is performed according to the obtained feature map. Finally, the two sets of features are spliced together. The first Ghost module in Figure 9(b) first reduces the number of output channels to 1/2 of the number of target output channels, and then the second Ghost module restores the number of channels to the number of target output channels and transmits the number of channels together with the residual. The incoming input feature maps are added point by point for feature fusion. As shown in Figure 9(c), use GhostBottleneck to replace all bottleneck modules in YOLOv5 and form a new GhostBottleneckCSP with the C3 module. The original bottleneck consists of 1 × 1 and 3 × 3 standard convolutions. The new structure replaces the original bottleneck. There are more 3 × 3 standard convolutions in the model, which reduces the amount of computation and compresses the model.

### 3.4. ShuffleConv

Most of the current excellent lightweight networks use group convolution or deep separable convolution to reduce the amount of computation generated by convolution operations. However, to achieve feature fusion between channels, the 1 × 1 convolution used in these networks takes up more computation throughout the process. To alleviate this problem, ShuffleNet [37] proposed the concept of channel mixing. After group convolution, the use of channel blending can realize the flow of information between groups and enhance the expression ability of features in a more economical way. Channel mixing can be achieved by conventional tensor operations, as shown in Figure 10.

The number in Figure 10 is the number of the input channels. The channel is extended to two dimensions using the reshape operation, and the extended two dimensions are replaced by transpose. Through this operation, the information between the group convolution channels can be fused without increasing the amount of computation. Finally, the flatten operation restores the two dimensions to the original initial dimension and completes the channel washing. Based on the above principle, it can be considered that a point-by-point convolution can be replaced by a 1 × 1 group convolution and a channel mixing operation combination. Compared with the standard convolution, the parameter number and calculation amount of the group convolution are greatly reduced, and the group convolution has a similar regular effect, which can reduce the probability of overfitting. For these advantages, this article improves the ordinary convolution operation in 6 Conv modules of 3 × 3 and 2 Conv modules of 1 × 1 in YOLOv5. The original ordinary convolution is replaced by group convolution and channel mixing module, which can theoretically realize further compression of the model.

### 3.5. Parameter Setting

#### 3.5.1. Loss Function

In the prediction of YOLOv5, Generalized IoU (GIoU) [38] is used as the loss function of BBox, and weighted nonmaximum suppression (NMS) is used. The loss function is shown in

(8) $$\begin{array}{c} L_{GIoU}=1-IoU+\frac{C-\left(B\cup B^{gt}\right)}{C}, \end{array}$$

(9) $$\begin{array}{c} IoU=\frac{A\cap B}{A\cup B}. \end{array}$$

However, when the prediction box is in the ground-truth box and the size of the prediction box is the same, the relative position of the prediction box and the ground-truth box cannot be distinguished.

Therefore, this article uses Complete IoU (CIoU) [39] to replace GIoU. Based on considering GIoU loss, CIoU loss considers the consistency of BBox overlapping area, center distance, and BBox aspect ratio. It can better predict the target. The definition of the loss function of GIoU is shown in

(10) $$\begin{array}{c} R_{CIoU}=\frac{\rho^{2}\left(b,b^{gt}\right)}{c^{2}}+\alpha \nu , \end{array}$$

(11) $$\begin{array}{c} \nu =\frac{4}{\pi^{2}}{\left(\arctan\frac{w^{gt}}{h^{gt}}-\arctan\frac{w}{h}\right)}^{2}, \end{array}$$

(12) $$\begin{array}{c} L_{CIoU}=1-IoU+R_{CIoU}, \end{array}$$

where *ρ*^2^(*b*, *b*^*gt*^) represents the Euclidean distance between the prediction box and the target box and *c*^2^ represents the diagonal distance of the minimum enclosing rectangle. *w*^*gt*^/*h*^*gt*^ and *w*/*h* represent the width-to-height ratios of the target box and the prediction box, respectively. The trade-off parameter is defined as *α*, which is a parameter greater than 0. The definition of trade-off parameters is shown in

(13) $$\begin{array}{c} \alpha =\frac{v}{\left(1-IoU\right)+v}. \end{array}$$

#### 3.5.2. K-Means ++ Clustering Anchor Frame

YOLOv5 conducts K-Means clustering on the COCO data set of general target detection and obtains the initial prior anchor frame. However, there are many types of targets in the COCO data set, which can reach more than 80 categories, and the types of pavement diseases in this article are 6 categories, which cannot meet the needs of actual disease detection. Therefore, it is necessary to redesign the size of the prior anchor frame. In this article, the K-Means ++ clustering algorithm is used to cluster the annotated target boundary anchor frames in the disease data many times, and different numbers and sizes of prior frames are generated as much as possible to increase the matching degree between the prior box and the actual target box, to further improve the detection accuracy. In the clustering process, the average intersection corresponding to the number of centers of different clusters is shown in Figure 11.

It can be seen from Figure 11 that when the number of prior frames is from 0 to 9, IoU shows a rapid upward trend, but when the number of prior frames is from 9 to 12, the growth rate of IoU slows down. In order to balance the detection accuracy and rate, nine prior anchor frames are finally selected, and the sizes of the anchor frames after clustering are, respectively, [54.2 99.2], [32.7 634.1], [604.1 354.2], [194.9 300.1], [251.2 95.9], [39.4 258.0], [47.1 427.7], [239.2 611.0], and [574.1 109.9]. The clustering center effect is shown in Figure 12.

### 3.6. FAFU-PD Data Set

Training a deep learning model with high accuracy and strong generalization ability needs to rely on large-scale and high-quality data sets, but many specific problems do not have a rich variety of public data sets, so it is particularly important to obtain high-definition pavement disease images. At present, the existing pavement disease data sets are collected by cameras installed in the cab or on the roof. In the actual highway inspection task, the image data collected in this way cannot well determine the pile number of the collection sites. There are two sources of road disease image data in this article: one is the road disease data provided by Fujian Highway Datong Detection Co., Ltd., and the other is the road disease data collected by the Digital Highway Data Vehicle (DHDV). As shown in Figure 13, the DHDV multifunction detection vehicle is jointly developed by Oklahoma State University, Arkansas University, and WAYLINK Company. The detection vehicle can collect road data at the speed of 100 km/h, and the acquisition range can cover a 4 m lane width. The accuracy of surface texture data collected in the vertical direction can reach 0.3 mm, and the accuracy of data in the longitudinal direction can reach 1 mm. The PaveVision3D sensor equipped on DHDV carries the latest imaging technology, which can obtain 2D and 3D laser imaging data from the road through two separate left and right sensors. Customized optical filters and high-power line laser projection systems enable DHDV to maintain consistency in image quality both during the day and night. DHDV collected part of the two-dimensional laser asphalt pavement nondeformation disease images as shown in Figure 14.

### 3.7. NST Algorithm

When detecting targets according to the characteristics of the object, the objects with similar characteristics are often classified as a class. Asphalt pavement disease is the target that we need to detect. In the actual detection process, it often conflicts with some other background targets. For example, the detection of crack diseases is often affected by the induction coil under the road, the lane scratch, and the pavement spray. The disease detection of patch type is often affected by pavement construction expansion joints, road markings, and indicator arrows. When the disease of patch type is detected, it is often affected by water stain, oil stain, and rutting. Particularly, when continuous water stain and oil stain occur on the pavement, the probability of false detection will be greatly improved.  Figure 15 shows the partial misdetection of the model.

To solve the hidden dangers brought by negative samples to road inspection, this article proposes a new negative sample training method. When training and labeling the target object, it is used as data for a series of backgrounds such as induction coils, water stains, and oil stains. The centralized negative sample labels, that is, the negative samples such as induction coils, water stains, and oil stains, are labeled. During the training process of the data set, the model will simultaneously label the positive samples (horizontal seam, vertical seam, patch, patch, etc.) and negative sample labels (induction coils, water and oil stains, etc.) for detection, and these negative sample labels can be excluded from the final detection results.

The advantages of this negative sample training method can be analyzed from the theory of information entropy. Information entropy is often used as a quantitative index of the information content of a system, which can be further used as the objective of system equation optimization or the criterion of parameter selection. The definition of information entropy is shown in

(14) $$\begin{array}{c} H\left(X\right)=-\sum_{i=1}^{n}p_{i}\log p_{i}, \end{array}$$

where*p*_*i*_ represents the probability that the *ith* symbol appears in the information source. *H* stands for information entropy.

After applying the NST method, positive sample (disease) tags and negative sample (background) tags may appear in the XML file generated by the detection. According to the principle of YOLOv5 and formula (14), the information entropy of the data set with and without negative sample labels can be obtained. From the principle of the neural network, it can be known that when the size of the image sent to the detection is different, it will affect the final recognition effect. We found that when the size of the image is 896, the number of false detections is converted into probability, before and after adding negative samples. The information entropy is 0.07405 and 0.07809, respectively; obviously, the gain is increased by 5.17%.

The negative samples and their labels of the NST method are shown in Figure 16.

### 3.8. Generative Adversarial Network Data Augmentation Algorithms

A generative adversarial network (GAN) is a game model based on adversarial generation proposed by Creswell et al. [40]. The GAN framework includes a generator network (*G*) and discriminator network (*D*). *G* and *D* confront each other through their respective strategies and reuse each other's strategies to adjust their strategies in time [41].

In our collected highway asphalt pavement disease data, the number of cracks, loose, and other diseases is small. To reduce the impact of unbalanced data types, we choose the GAN data enhancement algorithm to expand the amount of data on cracks, loose, and other diseases.

The basic framework of the GAN network used in this article is shown in Figure 17. The noise is fused into the original image to generate data. The generated data are input to *G* and the feature information of the pit is extracted. The fitting data are generated to deceive *D*, and *D* is used to identify the authenticity of the output data and feedback to the generated network to train the model.

Ratliff et al. [42] proposed Wasserstein distance to replace JS divergence (Jensen-Shannon divergence, JS), that is, Wasserstein generated adversarial network (WGAN) to improve the mode collapse problem of GAN. WGAN still has the problem of gradient explosion and gradient disappearance caused by gradient clipping. Therefore, Hsu et al. [43] proposed WGAN-GP with gradient penalty term. In this study, WGAN-GP with better data generation performance was used to generate pit data. The *G* and *D* of WGAN-GP were set to five layers of convolutional neural networks, and the number of layers was 1∼5. *G* is composed of transposed convolution (ConvTrans2d), batch norm (BN), and ReLu and Tanh activation functions. D is composed of convolution (Conv2d), instance norm (IN), and LeakyRelu activation functions. The detailed parameter settings of the network are shown in Table 4. In the table, *K* (kernel size, *K*) represents the size of the convolution kernel, *N*_out (number of out, *N*_out) represents the number of convolution kernels, and *S* (stride, *S*) represents the step size.

### 3.9. Poisson Migration Fusion Algorithm

In this study, the groove image generated by WGAN-GP is inserted into the disease-free road image to generate new training data. Firstly, the Poisson algorithm is used to output the fused image [44], and then the synthesized image is output by the color migration algorithm [45]. When integrating the image, the image should be integrated as real as possible. When synthesizing the image, the natural effect of the original data set should be maintained. Therefore, the color migration is added based on the Poisson fusion, which is called the Poisson migration fusion. As an image fusion method, the Poisson algorithm can better integrate the source image into the target image. In this study, the reference code of Poisson fusion implementation is shown in the literature. The color transfer algorithm can ensure that the target image and the reference image have the same pixel mean and variance in the color space. In this study, the color transfer implementation code is shown in the literature. In the Poisson algorithm, the pixel value of the unknown region is calculated by the Poisson equation, and the calculation method is shown in

(15) $$\begin{array}{c} \left\{\begin{array}{c} \underset{f}{\min}{\iint_{\omega }\left|\nabla f-v\right|}^{2}\\ f\left|\partial_{\omega }=f^{*}\right|\partial_{\omega }. \end{array}\right\}. \end{array}$$

Type: *ω* for the target image; ∇ is a gradient operator; *ν* is the gradient region in the image; *f* is the unknown function of the target image; *f*^*∗*^ is the known function of the source image; *∂*_*ω*_ is the boundary between the source image and the target image.

In the color transfer algorithm, the best matching pixel of the target image is found according to the color component of the reference image. The calculation method is shown in

(16) $$\begin{array}{c} T_{i,j}=\left|d_{i}-d_{j}\right|+\left|\sigma_{i}-\sigma_{j}\right|+\left|f_{i}-f_{j}\right|, \end{array}$$

where *i* and *j* are pixels of two images, respectively; *d*_*i*_ and *d*_*j*_ are the distance between pixels and clustering points; *σ*_*i*_ and *σ*_*j*_ are spatial dynamic selection coefficients of images; *f*_*i*_ and *f*_*j*_ are the average brightness of two images. The schematic diagram of the Poisson migration fusion algorithm is shown in Figure 18.

### 3.10. Softer-NMS

Softer-NMS for final result processing nonmaximum suppression (NMS) is mainly used for postprocessing of target detection model output based on deep learning, to remove redundant detection boxes and obtain correct detection results. But through the analysis we can find that NMS has the following defects:

- There are more missed detections in dense scenarios: when there is partial overlap between two targets nearer, there is a greater likelihood of missed detections for targets with less confidence.
- The NMS default box with higher confidence scores is more accurate, and this condition is not always valid because classification and regression tasks are not directly related. High confidence border boxes are not always more reliable than low confidence border boxes.
- The labeling of ground truth may not be reliable.

Aiming at the first problem of NMS, Soft-NMS designs the degree function of confidence score decline according to the size of IoU and has achieved certain results. But for the other two problems the classification confidence score is not strongly correlated with the IoU of the box, so a new method is needed to measure the location confidence of the box. Based on this, Softer-NMS puts forward two ideas, respectively, to build the confidence of IoU to model how much grasp that the current frame and GT are coincident; a method is proposed to combine multiple frames according to the IoU confidence to optimize the final generated frame. For IoU confidence, Softer-NMS uses Gaussian functions to model the prediction box. The calculation method is shown in

(17) $$\begin{array}{c} P_{\theta }\left(x\right)=\frac{1}{2\pi \sigma^{2}}e^{-{\left(x-x_{e}\right)}^{2}/2\sigma^{2}}. \end{array}$$

Using delta distribution to model GT frame, the calculation method is shown in

(18) $$\begin{array}{c} P_{D}\left(x\right)=\delta \left(x-x_{g}\right). \end{array}$$

In formulas (17) and (18), *P*_*θ*_(*x*) represents the Gaussian probability distribution of the predicted bounding box, *P*_*D*_(*x*) represents the delta probability distribution of the predicted bounding box, *x* represents the value of the actual bounding box, *σ* represents the standard deviation, *x*_*e*_ represents the prediction box after offset, and the output *x*_*g*_ represents the GT box.

Softer-NMS method can effectively avoid missed detection in complex asphalt pavement disease processing scenarios, to improve the recall rate and meet the needs of engineering tasks.

## 4. Experiments

### 4.1. Data and Experimental Environment

The experiment in this article requires good hardware configuration and GPU acceleration. The running environment of the experiment is shown in Table 5. The data set used in this article is from the subgrade and pavement safety detection platform of the Digital Fujian Intelligent Transportation Technology Internet of Things Laboratory of Fujian Agriculture and Forestry University and Fujian Expressway Datong Detection Company. This data set selects 7,000 training set images and 1750 test set images, respectively. To increase the robustness of the training model, the data set adds background images that do not contain diseases and adds background labels such as road markings, indicator arrows, and bridge joints. All label categories are shown in Table 6.

### 4.2. Ablation Experiment

#### 4.2.1. Evaluating Indicator

The automatic identification of highway asphalt pavement diseases belongs to the category of target detection. At present, the commonly used indexes to evaluate the training performance and robustness of the model are precision (P), recall (R), and mean average precision (mAP).

The target detection and evaluation index is applied to the test of highway asphalt pavement diseases, and two kinds of results images can be obtained, including images with diseases and images without diseases. True-positive (TP), false-positive (FP), true-negative (TN), and false-negative (FN) are important indicators to describe the accuracy of the model. The specific formulas of the above metrics are shown in

(19) $$\begin{array}{c} \text{Precision}=\frac{\text{TP}}{\text{TP}+\text{FP}}=\frac{\text{TP}}{\text{all detections}}, \end{array}$$

(20) $$\begin{array}{c} \text{Recall}=\frac{\text{TP}}{\text{TP}+\text{FN}}=\frac{\text{TP}}{\text{all ground truths}}, \end{array}$$

(21) $$\begin{array}{c} \text{AP}=\int_{0}^{1}P\text{d}R, \end{array}$$

(22) $$\begin{array}{c} \text{mAP}=\frac{\sum_{i=1}^{N}{\text{AP}}_{i}}{N}. \end{array}$$

TP, FP, and FN refer to correct check box, wrong check box, and missing check box, respectively. AP value is the area of the P-R curve, and N represents the total number of detection categories; this article is 10. mAP @ 0.5 refers to the average AP of all categories when IoU is set to 0.5. mAP @ 0.5 : 0.95 refers to the average mAP on different IoU thresholds. The IoU value ranges from 0.5 to 0.95, and the step length is 0.05. The average detection processing time includes network self-inference time and NMS processing time.

F1-score is a measure of classification problems. Some machine learning competitions for multiclassification problems often use F1-score as the final evaluation method. It is the harmonic average of precision rate and recall rate, with a maximum of 1 and a minimum of 0. Based on this, this article selects F1-score as the final model evaluation criteria. The calculation method of the F1-score is shown in

(23) $$\begin{array}{c} F_{1}=2\times \frac{\text{precision}\times \text{recall}}{\text{precision}+\text{recall}}. \end{array}$$

#### 4.2.2. Selection of Detection Image Size

In the process of image recognition, the larger the size of the image, the higher the clarity, the higher the recognition accuracy, and the slower the speed. The image with a small size is exactly the opposite. Therefore, how to balance the relationship between speed and accuracy is a very critical factor for us to select the image size. The variation trend of F1-score and FPS with the size of the detected image is shown in Figure 19. The black curve in the figure represents the change of the F1-score with the size of the detected image. The red curve represents the change of FPS with image size. It can be seen from the figure that the F1-score increases rapidly with the increase in image size. When the detection size exceeds 896, the curve becomes smooth. At the same time, the detection speed decreases with the increase of detection size. Considering this comprehensively, 896 is selected as the size of image detection, and 1024 is selected as the reference standard.

#### 4.2.3. Network Structure Ablation Experiment

In this section, the performance change caused by the change in network structure is gradually verified by ablation experiments. Four experiments are conducted for the target detection model of YOLOv5. Four networks, YOLOv5, YOLOv5-WPAN, YOLOv5-WPAN-Ghost, and YOLOv5-WPAN-Ghost-Shuffle (YOLO-W), are trained, respectively, in the four experiments. The network name can correspond to the structure described above one by one.  Figure 20 shows the precision curve of the four networks when the input image size is 896, and Figure 21 shows the recall curve of the four networks when the input image size is 896. The brightness of the curve increases in turn, respectively, representing YOLOv5, YOLOv5-W-PAN, YOLOv5-WPAN-Ghost, and YOLOv5-WPAN-Ghost-Shuffle (YOLO-W). In Figure 20, the accuracy of YOLOv5-WPAN-Ghost-Shuffle has an obvious loss, and the fluctuation is more intense. Fortunately, in the late training period, the difference between the accuracy of the model and YOLOv5 is lower than that in the early stage. The cause of fluctuations found during later debugging is related to batch-size settings.

As can be seen from Table 7, when the image size is 896, the calculation amount and parameters of the YOLOv5 network model with W-PAN structure are increased by 1.2% and 27.9%, respectively, and the F1-score is increased by 5.2%. After adding GhostBottleneck, the computation and parameters of the model are reduced to 53.3% and 65.3% of the original YOLOv5 network, respectively. The F1-score is increased by 7.5%, the model size is reduced by 37.8%, and the speed is increased by 5.9% with GPU.

After the standard convolution is replaced by ShuffleConv, the number of model parameters and the amount of calculation are further reduced to 29.5% and 29.3%, the F1-score is increased by 0.6%, and the model size is reduced by 29.9%. The result that the speed is not improved in the case of GPU is also expected. On the GPU platform with sufficient computing power, although the group convolution reduces the amount of computation and parameters, due to the limitation of memory exchange speed, the bottleneck of ShuffleConv is not the computational strength, so this module has little effect on the GPU environment. In addition, YOLOv5-WPAN-Ghost-Shuffle improves F1-score compared with YOLOv5-WPAN-Ghost, which proves the regularization effect of group convolution to some extent.

To further verify the efficiency of the proposed modules and networks, it is compared with similar lightweight networks YOLOv3-tiny and YOLOv4-tiny. It can be seen from Table 7 that the proposed network model has absolute advantages over YOLOv3-tiny and YOLOv4-tiny. The model size was only 59.0% and 44.7% of the above models, but the F1-score exceeded YOLOv3-tiny and YOLOv4-tiny by 13.6% and 10.6%. Therefore, the proposed model is reasonable and economical in engineering applications.

Secondly, by adding YOLOv3-tiny-Ghost-Shuffle, YOLOv3-tiny, YOLOv4-tiny-Ghost-Shuffle, and YOLOv4-tiny into two groups of comparative experiments, the optimization versatility of GhostBottleneck and ShuffleConv modules on other networks is proved. Compared with YOLOv3-tiny, YOLOv3-tiny-Ghost-Shuffle reduces the computation and parameter by 81.4% and 92.8%, respectively. The model size was compressed by 91.6% and the F1-score was increased by 1.4%. Compared with YOLOv4-tiny, YOLOv4-tiny-Ghost-Shuffle reduced the calculation amount and the number of parameters by 58.5% and 64.4%, respectively, reduced the model size by 58.5%, and increased the F1-score by 1.2%.

#### 4.2.4. GAN Ablation Experiment

In this section, we verify the performance change of the network model caused by the confrontational generation network (GAN) through ablation experiments. Three experiments are carried out for the YOLOv5 network model. The three experiments train YOLOv5, YOLOv5 + GAN + Poisson, and YOLO-W + GAN + Poisson networks, respectively. The experimental results are shown in Table 8. Taking the input image size of 896 as an example, YOLOv5 + GAN + Poisson is 2.54% higher than YOLOv5 in F1-score, and YOLO-W + GAN + Poisson is 9.13% higher than YOLOv5. Experiments show that the performance of the model can be effectively improved by adding a small number of diseases generated by the confrontation generation network (GAN) in the data set.

#### 4.2.5. NST Ablation Experiment

In this section, the data sets with and without nondisease labels are used for training, and the performance of each model in the NST ablation experiment is shown in Table 9. Taking the input image size of 896 as an example, YOLOv5+NST is 3.55% higher than YOLOv5 in F1-score, YOLOv5+GAN +Poisson+NST is 2.32% higher than YOLOv5+GAN+Poisson, and YOLO-W+GAN+Poisson+NST is 2% higher than YOLO-W+GAN+Poisson. Experiments show that the NST algorithm can effectively improve the performance of the model.

## 5. Analysis

To further verify the efficiency of the PDNet network architecture proposed in this article, the MMDetection tool is used to compare it with other classical networks on the FAFU-PD data set (including negative samples and generating disease data). These classical networks include a single-stage target detection network and a two-stage target detection network. The comparison results of different network performances are shown in Table 10.

The results show that this article improves the detection accuracy and speed of nondeformation diseases of asphalt pavement by improving the model network architecture design, parameter setting, and preprocessing algorithm. Combining our model with different processing techniques and using this as a comparison, our PDNet is essentially a YOLOv5-based nondeformable disease detection algorithm for asphalt pavements with additions such as Generative Adversarial Networks (GAN), Poisson transfer fusion algorithm, and negative sample algorithm (NST). The performance of the model is inseparable from the technology it adds. In the following, we will analyze the advantages of various processing techniques and how they work.

The W-PAN structure makes the fusion of semantic information at al levels of the network more reasonable and sufficient. The introduction of W-PAN has greatly improved the accuracy of the network, especially the accuracy of high-intersection which is higher than required. However, during its introduction also the parameter amount and calculation amount of the model are increased.

The addition of the Ghost module and Shuffle module reduces the computational complexity and parameter volume of the model and compresses the model.

Adversarial generative network (GAN) and Poisson transfer fusion algorithm generate disease types with a small number of samples, which solves the imbalance of training samples to a certain extent and improves the performance of the model without reducing the speed of the model.

The NST algorithm also improves the score without reducing the speed, because in the nondisease samples we increase the information entropy and increase the amount of useful information for disease detection.

In addition, the performance of the model is also affected by some parameter settings. For some parameters, some minor adjustments may cause the performance of the model to oscillate, such as the setting of the anchor box, the size of the detection image, and the number of detection layers.

Table 11 visually shows some performance differences of different types of models in the actual road test. From the YOLOv5 model to PDNet, the F1-score with detection sizes of 896 and 1024 is increased by 10.0% and 8.25% respectively; the speed of the model is increased by 15.5% FPS and 11.5 FPS to meet the needs of industrial applications.

## 6. Conclusion

In this study, based on the YOLOv5 target detection model, a real-time and high robustness detection network-PDNet for nondeformable diseases of asphalt pavement was realized. It realized the rapid and accurate detection of nondeformable diseases of asphalt pavement in the actual road detection process. When the image detection size was 896, the F1-score of 91.34 and the speed of 35.5 FPS were obtained on the Jetson nanoplatform. This algorithm will provide data support for the realization of highway daily maintenance. At the same time, the proposed W-PAN, GAN, Poisson, NST, and other technologies provide a reference for the specific application of artificial neural network optimization methods in edge computing equipment.

## Figures and Tables

**Figure 1:** Misrecognition or inaccurate recognition of deep learning models in engineering application scenarios: (a, b) target detection frame redundancy, (c, d) background is misidentified, (e, f) the target frame recognition is inaccurate, and (g, h) the disease characteristics are not obvious, and the detection is missed.

**Figure 2:** PDNet overall network framework. (a) Preprocessing side, (b) backbones, (c) necks, (d) heads, and (e) nondeformation disease detection of asphalt pavement.

**Figure 3:** The improved backbone module.

**Figure 4:** The improved neck module.

**Figure 5:** Schematic diagram of general feature fusion.

**Figure 6:** Schematic diagram of the cross-layer connection.

**Figure 7:** FPN structure used in this article (W-FPN).

**Figure 8:** Comparison of Ghost convolution and general convolution.

**Figure 9:** (a) Ghost module, (b) GhostBottleneck, and (c) GhostBottleneckCSP.

**Figure 10:** Experimental process of mixed washing in channels.

**Figure 11:** Number of centers of different clusters and average intersection-sum ratio.

**Figure 12:** Cluster center effect diagram.

**Figure 13:** DHDV multifunctional detection vehicle.

**Figure 14:** Two-dimensional laser asphalt pavement nondeformation disease image. (a) Repair-strip, (b) patch, (c) longitudinal crack, (d) crack, (e) transverse crack, and (f) loose.

**Figure 15:** Misdetection. (a) Misidentification of joints as a patch, (b) misidentification of lane markings as a patch, (c) misidentification of induction coils as transverse cracks, (d) misidentification of pavement scratches as longitudinal cracks, (e) misidentification of lane indicator arrows as patch, (f) misidentification of rut imprints as a patch, (g) misidentification of deceleration belts as patch, (h) misidentification of pavement splits as longitudinal cracks, and (i) misidentification of water stains as a patch.

**Figure 16:** Negative sample labels. (a) Expansion joints (joint), (b) road markings (laneMarking), (c) induction coils (coil), (d) lane scratches (scratches), (e) lane indication arrows (indicatesArrow), (f) rut, (g) speedBumps, (h) thrownObjects, and (i) waterStains.

**Figure 17:** Generating the basic framework of an adversarial network (GAN).

**Figure 18:** Schema of Poisson migration fusion algorithm.

**Figure 19:** F1-score and FPS versus image size.

**Figure 20:** Schematic diagram of the precision change curve.

**Figure 21:** Recall change curve diagram.

**Table 1:** YOLO-W algorithm architecture diagram.

Number	From	Parameters	Module
0	−1	3520	Focus
1	−1	10756	ShuffleConv
2	−1	10016	GhostC3
3	−1	40868	ShuffleConv
4	−1	41840	GhostC3
5	−1	159460	ShuffleConv
6	−1	173304	GhostC3
7	−1	466468	ShuffleConv
8	−1	325016	GhostC3
9	−1	925028	ShuffleConv
10	−1	656896	SPP
11	−1	575112	GhostC3
12	−1	103872	ShuffleConv
13	−1	0	Upsample
14	[−1, 8]	0	Concat
15	−1	466512	GhostC3
16	−1	52864	ShuffleConv
17	−1	0	Upsample
18	[−1, 6]	0	Concat
19	−1	208608	GhostC3
20	−1	18240	ShuffleConv
21	−1	0	Upsample
22	[−1, 4]	0	Concat
23	−1	53104	GhostC3
24	−1	75584	ShuffleConv
25	[−1, 20]	0	Concat
26	[−1, 6]	36482	Add
27	−1	143072	GhostC3
28	−1	298624	ShuffleConv
29	[−1, 6]	0	Concat
30	[−1, 8]	105730	Add
31	−1	368208	GhostC3
32	−1	669120	ShuffleConv
33	[−1, 12]	0	Concat
34	−1	695744	GhostC3
35	[23, 27, 31, 34]	96300	Detect

**Table 2:** Comparison of YOLOv5s effects before and after deepening the pyramid.

Module	Parameters	GFLOPs	F1-score (%)
PAN	7114785	16.5	81.34
W-PAN-Deep	12395500	16.7	84.39

**Table 3:** Comparison of the effects of W-PAN-Deep and PAN under YOLOv5s.

Module	F1-score (%)
PAN	81.34
W-PAN-Deep	84.39
W-PAN	85.77

**Table 4:** WGAN-GP network detailed parameter table.

Layers	Net	Parameters
G1	ConvTrans2d + BN + ReLu	*K*: 4, *N*_out : 512, *S*: 1
G2	ConvTrans2d + BN + ReLu	*K*: 3, *N*_out : 256, *S* : 2
G3	ConvTrans2d + BN + ReLu	*K*: 3, *N*_out : 128, *S*: 3
G4	ConvTrans2d + BN + ReLu	*K*: 4, *N*_out : 64, *S*: 4
G5	ConvTrans2d + Tanh	*K*: 6, *N*_out : 64, *S*: 4
D1	Conv2d + IN + LeakyReLu	*K*: 6,*N*_out : 64,*S*: 4
D2	Conv2d + IN + LeakyReLu	*K*: 4, *N*_out : 64, *S*: 4
D3	Conv2d + IN + LeakyReLu	*K*: 3, *N*_out : 128, *S*: 3
D4	Conv2d + IN + LeakyReLu	*K*: 3, *N*_out : 256, *S*: 2
D5	Conv2d	*K*: 4, *N*_out : 512, *S* 1

**Table 5:** Experimental operational environment.

Category	Entry	Version
Hardware configuration	System	Windows 10

Software configuration	Graphics card CPU	GeForce RTX 3080 Intel(R) core(TM) i7-6700 CPU
	Python version	3.8
	Deep learning framework	PyTorch
	CUDA	10.0

**Table 6:** All label categories in the data set.

Disease	Label	Nondisease	Label
Transverse crack	TransverseCrack	Deck expansion joint	Joint
Longitudinal crack	LongitudinalCrack	Road marking	LaneMarking
Alligator crack	AlligatorCrack	Induction coil	Coil
Repair-strips	Sealing	Scratch	Scratches
Repair block	Patch	Guide finger	IndicatesArrow
Loose	Loose	Rut	Rut
Repair seam	SealingCrack	Deceleration strip	SpeedBumps
		Sprinkler	ThrownObjects
		Water stain	WaterStains

**Table 7:** Performance comparison of models in network structure ablation experiment.

Size	Model	Parameters	GFLOPS	Speed-GPU	Weight	F1-score (%)
896	YOLOv5	7114785	16.5	1.7	14.2	81.34
	YOLOv5-WPAN	9874167	16.7	1.9	15.6	85.77
	YOLOv5-WPAN-Ghost	3419817	7.8	1.6	9.7	87.97
	YOLOv5-WPAN-Ghost-Shuffle	2419191	5.5	1.6	6.8	88.49
	YOLOv3-tiny	8669002	12.9	1.7	16.6	76.44
	YOLOv3-tiny-Ghost-Shuffle	620344	2.4	2.3	1.4	77.56
	YOLOv4-tiny	6399178	21.8	1.9	12.3	79.13
	YOLOv4-tiny-Ghost-Shuffle	2278010	8.4	1.9	5.1	80.11

1024	YOLOv5	9347865	16.7	1.6	17.8	84.13
	YOLOv5-WPAN	11934134	16.9	1.8	19.1	86.14
	YOLOv5-WPAN-Ghost	4321786	8.4	1.8	7.4	88.03
	YOLOv5-WPAN-Ghost-Shuffle	3376145	6.3	1.2	5.4	89.32
	YOLOv3-tiny	9478945	13.1	1.5	18.7	77.44
	YOLOv3-tiny-Ghost-Shuffle	6945879	3.7	2.1	2.9	79.56
	YOLOv4-tiny	7456849	22.3	1.7	6.8	80.99
	YOLOv4-tiny-Ghost-Shuffle	3415684	10.4	1.7	7.5	81.46

**Table 8:** Performance comparison of GAN ablation models.

Size	Model	F1-score (%)
896	YOLOv5	81.34
	YOLOv5 + GAN + Poisson	83.46
	YOLO-W + GAN + Poisson	89.51

1024	YOLOv5	84.13
	YOLOv5 + GAN + Poisson	84.55
	YOLO-W + GAN + Poisson	90.74

**Table 9:** Performance comparison of NST ablation models.

Detection size	Model	Training set classes	F1-score (%)
896	YOLOv5	Disease	81.34
	YOLOv5 + NST	Disease + nondisease	84.33
	YOLOv5 + GAN + Poisson	Disease	83.46
	YOLOv5 + GAN + Poisson + NST	Disease + nondisease	85.44
	YOLO-W + GAN + Poisson	Disease	89.51
	YOLO-W + GAN + Poisson + NST	Disease + nondisease	91.34

1024	YOLOv5	Disease	84.13
	YOLOv5 + NST	Disease + nondisease	84.33
	YOLOv5 + GAN + Poisson	Disease	84.55
	YOLOv5 + GAN + Poisson + NST	Disease + nondisease	86.74
	YOLO-W + GAN + Poisson	Disease	90.74
	YOLO-W + GAN + Poisson + NST	Disease + nondisease	92.38

**Table 10:** Performance comparison table of different network models.

Methods	Backbone	F1-score (%)
*Two-stage*		
Faster R-CNN	Resnext101	75.14
Cascade R-CNN	Resnext101	75.17
Libra R-CNN	Resnext101	76.33
Grid R-CNN	Resnext101	76.22
Mask R-CNN	Resnext101	76.22
Dynamic R-CNN	Resnet50	76.23

*One-stage*		
FCOS	Resnext101	76.13
FreeAnchor	Resnext101	76.13
RepPoints	Resnext101	76.12
PAA	Resnext101	76.32
ATSS	Resnet101	75.11
FoveaBox	Resnet101	74.36
FSAF	Resnext101	76.12
VFNet	Resnext101	76.11
SSD512	Vgg16	75.33
RetinaNet	Resnext101	76.46
YOLOv3	CSPdarknet	76.47
YOLOv4	CSPdarknet	79.33
YOLOv5s	CSPdarknet	81.34
Ours	Ours	91.34

**Table 11:** Performance parameters of each model in the actual test section.

Model	896		1024	
	Speed (FPS)	F1-score (%)	Speed (FPS)	F1-score (%)
YOLOv5	20.0	81.34	5.2	84.13
YOLO-W	33.5	88.49	16.0	89.32
YOLO-W + GAN + Poisson	35.5	89.51	16.1	90.74
YOLO-W + GAN + Poisson + NST(PDNet)	35.5	91.34	16.7	92.38

## Data Availability

The data used to support the findings of this study are included within the article.
